# Oculomotor Guidance and Capture by Irrelevant Faces

**DOI:** 10.1371/journal.pone.0034598

**Published:** 2012-04-10

**Authors:** Christel Devue, Artem V. Belopolsky, Jan Theeuwes

**Affiliations:** 1 Cognitive Psychology, Vrije Universiteit Amsterdam, Amsterdam, The Netherlands; 2 Department of Psychology, Cognition and Behavior, Université de Liège, Liege, Belgium; Kyushu University, Japan

## Abstract

Even though it is generally agreed that face stimuli constitute a special class of stimuli, which are treated preferentially by our visual system, it remains unclear whether faces can capture attention in a stimulus-driven manner. Moreover, there is a long-standing debate regarding the mechanism underlying the preferential bias of selecting faces. Some claim that faces constitute a set of special low-level features to which our visual system is tuned; others claim that the visual system is capable of extracting the meaning of faces very rapidly, driving attentional selection. Those debates continue because many studies contain methodological peculiarities and manipulations that prevent a definitive conclusion. Here, we present a new visual search task in which observers had to make a saccade to a uniquely colored circle while completely irrelevant objects were also present in the visual field. The results indicate that faces capture and guide the eyes more than other animated objects and that our visual system is not only tuned to the low-level features that make up a face but also to its meaning.

## Introduction

In everyday life, we constantly look around and use our visual input to guide our behavior. When search is controlled by our intentions and goals, one speaks of top-down, goal-directed selection. However while searching for a particular object, we may sometimes attend to things in our environment which we had no intention to look for. In that case, our selection is captured by the features in the environment in a bottom-up, stimulus driven manner (see [1], [2] for reviews). While it has been demonstrated often that stimuli such as abrupt onset flashes or unique colors may capture our attention [3] or even our eyes [4] in a bottom-up fashion, it is unclear whether this also holds for stimuli that have high socio-biological value and relevance, such as the human face. Human faces convey a wealth of information relevant to our social lives (e.g. identity, gender, age, ethnic origin, emotions or intentions of our fellow humans) and it is of crucial importance to access this information as promptly as possible. Since faces all have the same basic structure and face information is coded in dedicated brain areas (e.g. fusiform face area; see e.g. [5], [6]; but see e.g. [7]), it may not be surprising that faces can be detected very efficiently. Even though plausible, the current literature does not provide a clear and coherent picture whether the selection of human faces really occurs in a stimulus-driven fashion (see e.g. [8] for a review). Besides, the relative contribution of low-level features constituting a face or of the meaning conveyed by faces in possible capture effects is also highly debated. Some data suggests that faces contain low-level features to which our visual system is tuned (see e.g. [9]) while others indicate that the visual system can quickly extract the meaning of faces, driving attentional selection (see e.g. [10]).

A variety of paradigms have shown attentional biases towards faces. Upright faces seem to be more resistant to attentional blink [11] (but see [12]), to change blindness [13]–[15] (but see [16], [17]), to inattentional blindness [18], [19] and they produce inhibition of return [20] by comparison with other objects or inverted faces. In addition, faces are less likely to be extinguished in patients with visual neglect [21]. Also studies using visual search in which faces and other objects have to be detected provided mixed results. Some studies reported a pop-out effect for faces [22], [23] while others did not (e.g. [9], [24]). From results of this type of paradigm, some claim that faces capture attention in a bottom-up way [10], [14] but the relative contribution of bottom-up and top-down factors is actually difficult to distinguish in such search tasks because people are intentionally looking for task-relevant faces.

Therefore, while some data seem to indicate that faces attract attention, they do not unequivocally show that it is due to a bottom-up capture. Rather, they could be due to our high expertise with faces leading them to be easier to process than other stimuli when the task requires a detection or a categorization of the stimuli or to difficulties in disengaging attention from faces once they are attended [25] possibly pointing out to a mere preference for facial stimuli. Furthermore, some studies have also shown that faces can be ignored when they are presented as distractors in more complex visual displays [26] (see also [27]), indicating that their processing is not mandatory.

To circumvent the interpretation issue in terms of the ability of faces to capture attention in a bottom-up manner, a new task was developed which involved an oculomotor version of a capture task (cf. [4]). Participants had to make a saccadic eye movement while a face was present in the display. Crucially, to assess pure bottom-up selection, we ensured that the critical stimulus was completely irrelevant for the task at hand. If in those circumstances the critical stimulus is selected first one can speak of bottom-up capture [2], [28]. Moreover, we were also willing to assess the relative contribution of the meaning conveyed by faces and of low-level features contained in faces in case of bottom-up capture. To that purpose, we compared the effect of faces that were presented upright to that of faces presented inverted (see e.g. [10]).

Participants searched for a uniquely colored circle and had to make a saccade to that color singleton target while six other completely irrelevant objects were present in the display (see Figure 1). We examined the effect of the presence of three types of irrelevant objects (a face, an inverted face and a butterfly) presented during different trials on eye movement behavior. We used a butterfly as control stimulus by analogy with what had been done in a previous study by Langton and colleagues [10] and in order to compare the effect of three types of living objects presented among inanimate objects (i.e. the five other objects the display consisted of). The location of these critical objects coincided with the location of the color singleton target at chance level, so there was no incentive to attend to them. On trials when the location of the critical object did not coincide with the location of the target, we assessed whether these stimuli could capture the eye (i.e., oculomotor capture). If faces have the ability to capture the eyes, we expect more capture when a face is present than when a critical control stimulus is present (in this case, a butterfly). Critically, if it is not only the low-level features of a face that captures the eyes, but also its meaning as a face, we expect more oculomotor capture for an upright canonical face than for an inverted face. Furthermore, our design made it possible to also examine the oculomotor guidance on trials in which the critical object happened next to the target. If it is the meaningfulness of the face that is prioritized for selection, one expects to find a greater facilitation of eye movements for trials with an upright face than for those with an inverted face. However, if faces are prioritized only because of the salience of their low-level features then both upright and inverted faces should guide the eyes in their direction equally strongly.

**Figure 1:** Illustration of a display used in the present study. Participants were instructed to make a saccade to a unique colored target circle and ignore the pictures of objects. Here, an upright face is presented as critical object and its spatial location mismatches that of the target (orange circle).

## Methods

### Participants

Twenty four students participated (6 males; mean age=23.54 years, SD=3.78). The present study was approved by the ethics board of the Faculty of Psychology and Education (VCWE) at the Vrije Universiteit Amsterdam and was conducted according to the Declaration of Helsinki. All the participants signed an informed consent before being included in the study. They received course credits or money for their participation.

### Stimuli and displays

Each display consisted of 6 grayscale pictures of objects (at 6.3° of eccentricity) surrounded by 6 colored circles (diameter=1 degree, at 8.7° of eccentricity). There were one object of interest (i.e., upright face, inverted face or butterfly; hereafter called “critical object") and 5 other objects. There were nine categories of pictures, each one having 8 exemplars, so that a total of 72 pictures were used. Faces were frontal view pictures of 4 male and 4 female models displaying a neutral facial expression. Hair below the ear lobes and neck were removed so that all faces had an overall oval shape but also a natural appearance. Inverted faces were created by flipping the pictures vertically. In addition, there were 6 categories of inanimate objects used as filler items, i.e. clothes, dishes, domestic devices, musical instruments, toys and vegetables. They were chosen to be visually different from both faces and butterflies but also from each other, while belonging to clear categories. Each picture was cropped and resized to fit within approximately 2.4° square. The circles surrounding those objects all had the same color (i.e. green or orange) except one that had a different color (i.e. orange or green) and constituted the target. For each trial, the combination of colors was chosen at random.

### Procedure

Participants were tested individually in a dim-lighted room on a PC. They were sited at a 75 cm distance, controlled by means of a chin-rest, from a 17-inch monitor with a 1024×768 resolution. Eye movements were measured with an Eye Link II eye tracking system with 500 Hz sampling rate. An automatic algorithm detected saccades using minimum velocity and acceleration criteria of 35°/s and 9,500°/s^2^ respectively.

Participants had to make a saccade to the uniquely colored target circle as fast and accurately as possible. They were informed that the objects were totally irrelevant to the correct realization of the task and instructed to ignore them. Each trial began with a drift correction screen triggered by a space bar press from the participant while fixating at a central fixation cross. The fixation cross subsequently stayed on for a duration varying randomly between 600 and 1000 ms to prevent anticipatory eye movements. A blank screen was then presented for 200 ms to ease attentional disengagement from fixation before the appearance of the search display. The display was presented for 1000 ms and was followed by a 500 ms blank screen. Participants received a high tone sound as auditory feedback in case of anticipatory saccade (i.e. before the display onset) and a low tone sound in case of too slow response (i.e. eyes still within the central area 600 ms after the display onset).

There were 1080 trials (i.e. 20 blocks of 54 trials interrupted by breaks). Each critical object (i.e. upright face, inverted face and butterfly) appeared within the display in a third of the trials. The categories of the 5 filler items were picked out at random among the 6 possible categories and the items presented were randomly picked out among the 8 possible exemplars of their category. The positions of the target circle and of each type of critical object relative to the target were counterbalanced across the trials, resulting in 60 trials in which their spatial locations matched and 300 trials in which their positions did not match. So for each of the 6 possible positions of the target, each type of critical object appeared 10 times at each of the 5 remaining locations. This was to ensure that the position of a critical object was totally non-predictive of the position of the target circle.

### Design and data analysis

We examined oculomotor capture: how often did the eyes go inadvertently to the critical object. In addition we analyzed oculomotor guidance (i.e., critical object presented next to the target circle [match trials]) and interference (i.e. critical object presented at another location than the target [mismatch trials]) on saccadic latency, accuracy, search time, and number of saccades necessary to reach the target. For these data we reported the critical 2-way Match×Critical Object interactions and conducted planned comparisons assessing the effect of the spatial location for each type of critical object. To compare the impact of upright and inverted faces we conducted a follow-up analysis to test for 2-way Match×Face type interaction.

Trials with anticipatory (first saccade latency <80 ms after the display onset) or late (first saccade latency >600 ms) saccades were excluded from the analyses (i.e. 4% of trials). We defined a saccade as going in the direction of one of the six circles/objects when the saccadic endpoint lied within 30° of arc on either side of the centre of the target.

## Results

### Oculomotor capture

We conducted a one-way ANOVA with Critical Object type as factor on the percentage of trials in which the eyes went first to the critical object during mismatch trials (see Figure 2A). There was a significant effect of Critical Object type, *F*(2,46)=22.46; *p*<0.001. Planned comparisons showed that upright faces (*M*=13.12%, *SD*=5.94) captured the eyes more than inverted faces (*M*=10.8%, *SD*=4.33), *p*<0.01, and butterflies (*M*=8.5%, *SD*=3.7), *p*<0.001. Inverted faces also captured the eyes more than butterflies, *p*<0.001. When oculomotor capture occurred, we also analyzed the time the eyes remained fixated at the critical object (Figure 2B). We only found a marginal effect of Critical Object type, *F*(2,46)=2.54; *p*=0.089. This absence of reliable effect might be due to a lack of power because this measure was only possible on a limited amount of trials (i.e., between 8.5 and 13.12% of mismatch trials, that is about 24.5 to 38 trials). We thus conducted planned comparisons to test the a priori hypothesis that upright faces might retain the eyes longer than the other types of critical objects. They showed that upright faces (*M*=108.9 ms; *SD*=25.3) were fixated longer than butterflies (*M*=101.2 ms; *SD*=20.6), *p*<0.05 (see Figure 2B). Other comparisons did not reach significance (*p*s>0.12).

**Figure 2:** Influence of the Critical object type during mismatch trials. Mean percentage of oculomotor capture (A) and mean fixation durations following oculomotor capture (B). Error bars represent 95% confidence intervals (CI; see [29]).

### Oculomotor guidance

If the eyes get captured by the critical object, there should also be a benefit when the target circle is close to the critical object. We examined the interaction between the Critical Object type (upright face, inverted face, butterfly) and its location in the visual field (match: next to the target circle; vs. mismatch: somewhere else in the display). Figure 3 presents the results. With respect to latency, there was an interaction between Critical Object type and Match, *F*(2, 46)=6.58; *p*<0.005, showing that only in case of upright faces, but not for the two other critical objects (both *p*s>0.15), participants were faster in making a saccade to the matching target circle than to a mismatching target, *p*<0.001. A follow-up Match×Face type (upright vs. inverted) ANOVA also revealed a significant interaction, *F*(1, 23)=4.46; *p*<0.05, indicating that upright faces had a larger effect on latency than inverted faces (see Figure 3A). Regarding accuracy, the interaction between Critical Object and Match was also significant, *F*(2,46)=7.13; *p*<0.005, with a higher accuracy for matching than for mismatching trials for upright, *p*<0.001, and inverted faces, *p*<0.005, but not for butterflies, p=0.7. Here again, a follow-up ANOVA revealed a significant interaction between Match and Face type, *F*(1, 23)=4.49; p<0.05 (see Figure 3B). For search time the interaction between Critical Object and Match was also reliable, *F*(2,46)=12.02; *p*<0.001, with faster search times for matching than for mismatching trials for upright and inverted faces, *p*<0.001 and *p*<0.05, respectively, but not for butterflies, *p*=0.89. Upright faces had a larger impact on the search time than inverted faces, as revealed by a significant Match×Face type interaction, *F*(1, 23)=7.96, *p*<0.01 (see Figure 3C). For the number of saccades the critical interaction between Match and Critical Object type was also reliable, *F*(2,46)=6.86; *p*<0.005, with an upright face significantly reducing the number of saccades during match trials relative to mismatch trials (*p*<0.001). Inverted faces only tended to do so, *p*=0.071, while the location of butterflies had no effect, *p*=0.88. The follow-up Match×Face type interaction was also significant, *F*(1, 23)=7.53; *p*<0.02, suggesting that the impact of upright faces upon the number of saccades was greater than that of inverted faces (see Figure 3D).

**Figure 3:** Oculomotor guidance and interference by the different Critical objects. Results of the search task in terms of mean latency (A), mean accuracy (B), mean search time (C) and mean number of saccades to reach the target (D), as a function of the critical object type included in the display and as a function of the location of the critical object matching or not that of the target. Error bars represent CI.

## Discussion

The results indicate that the presence of an irrelevant face somewhere in the visual scene has an effect on oculomotor behavior. Our results suggest a bottom-up oculomotor capture by an upright face and to a lesser extent by an inverted face. When it captured the eyes, the upright face also tended to hold the eyes a bit longer.

The presence of an upright face had also an effect on the oculomotor guidance as evidenced by all of our measures (Figure 3). It disrupted the search when it was located away from the target and guided the search when located next to the target. Importantly, inverted faces had a similar but less robust effect on the oculomotor behavior, suggesting that low-level features of the face also have the ability to affect selection in a bottom-up way. Finally, the presence of the neutral object (i.e., the butterfly) had no effect on oculomotor behavior as the pattern of results was similar whether a butterfly was located next to or away from the target.

These present findings provide a very coherent picture. Consistent with previous studies we show that face stimuli are prioritized by our visual system by comparison with other animated objects (e.g. [10], [15], [22], [23]). More importantly however this prioritization is not necessarily the result of some top-down preference to look at face stimuli (e.g. [14]) but seems to occur in a bottom-up stimulus-driven manner (e.g. [10]). Even though the task we used was very easy (i.e., make a saccade to the color singleton) and the target singleton can be detected by parallel processing participants could not always ignore the completely irrelevant pictures of objects. Our data show that the effect is partly due to low-level feature characteristics of the face stimuli, as the effects are also seen for inverted faces (e.g. [30]). However, on top of this, an upright face has both a stronger effect on guidance and capture than inverted faces, suggesting that the visual system is not only tuned to the low-level features that make up a face (salience) but also to the meaning (semantics) of a face. Finally, an upright face also seems to hold the eyes longer than non-face stimuli (see also [15]). By measuring eye movement behavior we have thus provided indications as to the processes at play when a task-irrelevant facial stimulus interferes with an ongoing task and as to a cumulative contribution of low- and high-level features.

One might object that, despite the fact that their spatial location was totally unpredictive of the color singleton target, participants might have interpreted an experimental demand to attend to upright and inverted faces given that they were distinctive stimuli among the rest of the set and that a similar advantage might have been afforded to any anomalous stimulus. However, if this would be the case, one should have expected inverted faces to attract the eyes even more than upright faces since inverted faces constituted a more abnormal stimulus (i.e. they were the only stimulus to appear upside down), which was in fact not the case.

Since faces seem to capture attention and drive the oculomotor system very early on, we might assume that faces (and not just their low-level features but their actual meaning) are detected preattentively, attract attention automatically, and then cause the eyes to move towards them. When participants are required to make a goal-directed saccade towards the colored target circle, the reflexive shift of attention towards the face causes the programming and possible execution of a stimulus-driven saccade towards the face. The mechanism underlying these effects is presumably identical to those described in oculomotor capture with an abrupt onset as a distractor [4], [31]. According to the competitive integration model [32] goal-directed and stimulus-driven saccades are programmed in a competitive way in a common saccade map. Note that it remains possible that this early detection of facial features leading to bottom-up capture might depend upon the complexity of the visual environment in which a face appears. Such a capture by task-irrelevant faces could have had not occurred in cases where insufficient attentional resources were available to process them, as indicated in the studies by Bindemann and colleagues [26], [27]. Our rationale here was to compare the ability of faces and of non-face objects to attract the eyes in contradiction with the task requirements, which we interpreted as an automatic capture (see [4]). The extent of this ability of faces to attract the eyes automatically could be tested further in future studies by manipulating the complexity of the environment.

The assumption of an early preattentive detection of a face among other competing objects is nonetheless consistent with other studies that have suggested that faces are encoded preattentively (e.g. [10], [20], [33]). Moreover, the results are also consistent with recent finding of Kirchner and Thorpe [34] (see also [35]) who showed, by means of a forced-choice saccade task, that people can categorize natural scenes very quickly. For example, when viewing two scenes, participants could reliably make saccades to the one containing an animal in as little as 120 ms. Low-level differences between target and distractor images could not explain these remarkably fast responses, suggesting that the meaning of animate objects can be derived very quickly, in such a way that it affects the programming of eye-movements.

In everyday life, particular objects or events may catch our eye even when we have other intentions. The current study shows that the presence of a face in our environment may interrupt our goal-directed eye movement behavior and grab our eyes more than other types of animated objects. Such a mechanism may be ecologically beneficial because finding other humans is important to us.
